# Weight loss reduces breast ductal fluid estrogens in obese postmenopausal women: a single arm intervention pilot study

**DOI:** 10.1186/1475-2891-11-102

**Published:** 2012-12-05

**Authors:** Catherine L Carpenter, Karen Duvall, Patricia Jardack, Luyi Li, Susanne M Henning, Zhaoping Li, David Heber

**Affiliations:** 1 Center for Human Nutrition, David Geffen School of Medicine at UCLA, Los Angeles, CA, USA; 2 School of Nursing, University of California at Los Angeles, Los Angeles, CA, USA; 3 Center for Health Promotion and Disease Prevention; David Geffen School of Medicine, University of California at Los Angeles, Los Angeles, CA, USA; 4 General Clinical Research Center; David Geffen School of Medicine, University of California at Los Angeles, Los Angeles, CA, USA

**Keywords:** Obesity, Postmenopausal, Diet, Exercise, Breast cancer, Breast ductal fluid

## Abstract

**Background:**

Accumulation of excess body fat increases breast cancer risk after menopause. Whether the localized breast is differently influenced by adipose tissue compared to the rest of the body, has not been well studied. Our purpose was to demonstrate feasibility and preliminarily evaluate serum-based and localized breast biomarker changes resulting from a weight loss intervention among obese postmenopausal women.

**Methods:**

We conducted a 12-week pilot controlled dietary and exercise intervention among healthy obese postmenopausal women, collected serum and breast ductal fluid before and after the intervention, and estimated the association with systemic and localized biomarker changes. We recruited 7 obese (mean body mass index = 33.6 kg/m^2^) postmenopausal women. We collected samples at baseline and the 12th week for: anthropometry; phlebotomy; dual-energy x-ray absorptiometry (lean and fat mass); exercise fitness (maximum oxygen consumption (VO_2_Max); 1-repetition strength maximum); and breast ductal lavage.

**Results:**

Changes from baseline occurred in body composition and exercise performance including fat mass loss (14% average drop), VO_2_Max (+36% increase) and strength improvement (+26%). Breast ductal fluid markers declined from baseline with estradiol showing a 24% reduction and IL-6 a 20% reduction. We also observed serum biomarker reductions from baseline including leptin (36% decline), estrone sulfate (−10%), estradiol (−25%), and Il-6 (−33%).

**Conclusions:**

Conduct of the diet and exercise intervention, collection of ductal fluid, and measurement of hormones and cytokines contained in the ductal fluid were all feasible. We preliminarily demonstrated estradiol and IL-6 reductions from baseline in both serum and breast ductal fluid among obese postmenopausal women who participated in the 12-week weight loss diet and exercise intervention.

## Background

The rising obesity prevalence and resulting increase in adipose tissue derived factors provide a strong rationale for developing effective weight-loss interventions. The majority of diet and exercise interventions designed for breast cancer prevention are targeted toward systemic parameters. However evidence suggests that the localized breast environment may be exposed to higher levels of adipose-derived hormones, cytokines, and inflammatory factors [1].

Most invasive breast cancers originate in terminal duct lobular units consisting of ducts that travel from the openings located on the nipple-areola complex into the breast parenchyma [2]. While hormones during each menstrual cycle affect proliferation of ductal cells and their differentiation [3], after menopause there is an involution of the ducts and alveoli in the breast [4]. Surrounding fibrous connective tissue change in density and breast tissues are replaced by adipose tissue. Fluid derived from lymphatic tissue travels in the non-lactating breast ducts and can be non-invasively obtained from nipple aspiration and ductal lavage procedures [5]. Ductal fluid has been shown in early studies to contain hormones, growth factors, environmental contaminants, and dietary metabolites [6-9].

Adulthood weight gain and obesity increase breast cancer risk after menopause [10-13]. Several possible mechanisms link body fat to breast cancer risk including oxidative stress [14], inflammation from abdominally distributed body fat [15,16], and excess estrogen production [17]. These mechanisms can function locally depending on the distribution of body fat and systemically in terms of body fat production of hormones and cytokines that travel in plasma.

The breast environment can be the recipient of both serum-based and locally derived hormones and inflammatory cytokines. Fat tissue surrounding the stroma and ductal epithelium, for instance, has particularly high levels of aromatase enzyme activity [18,19]. Enhanced localized aromatase activity coupled with estradiol levels in the circulating plasma can potentially deliver a more potent dose of estradiol to the localized breast than the rest of the body.

Localized breast measurements may be critical to evaluating risk reduction strategies. Diet and exercise has been shown in multiple studies to protectively impact serum-based estrogen, inflammation and oxidative stress biomarkers [20-23]; however, sparse data exists for more localized effects on the breast. Collection of breast ductal fluid could provide a medium of localized concentration of risk and preventive biomarkers such as dietary micronutrients, cytokines, and hormones found in the breast. Several recent studies detected inflammatory cytokines, markers of oxidative stress, and hormones in nipple aspirate, breast milk, and breast ductal fluid [24-28].

In order to establish feasibility and preliminarily estimate the association between the controlled feeding and exercise intervention on serum-based and localized breast biomarkers, we conducted a 12-week pilot study among obese sedentary postmenopausal women. We drew blood samples to measure systemic hormonal and cytokine markers, collected breast ductal fluid before and after the intervention, and evaluated change in breast biomarkers contained in the ductal fluid.

## Methods

### Study design and recruitment

A single 12-week intervention was conducted among obese sedentary postmenopausal women recruited from two sources: research staff working at UCLA and the Love/Avon Army of Women. Eligibility criteria included not having had menses for two or more years, age less than 75 years old, being sedentary (undergoing less than 1 hour per week of moderate or vigorous intensity recreational exercise), and having a body-mass-index (BMI) between 25.0 kg/m^2^ and 35 kg/m^2^. We excluded women who could not physically undergo the exercise intervention, women currently on a weight loss program, women who ever had weight reduction surgery, or women consuming more than 3 servings of fruits and vegetables per day (to eliminate participants likely to consume healthy diets). We set an upper BMI limit of 35.0 kg/m^2^ to ensure women would not be too heavy to undergo the exercise intervention.

We utilized two sources of subjects: UCLA staff members and the Love/Avon Army of Women. We posted flyers around the UCLA campus inviting eligible women to participate, and a call was put out to the Army of Women (see reference #29) in early 2009 [29]. A total of 50 women were interested in participating (25 from UCLA and 25 from the Love/Avon Army of Women), and all were screened over the telephone. Of the 50 women, 13 were ineligible, 3 changed their minds, and 26 were not able to fully participate. Five women from UCLA and 3 women from the Love/Avon Army of Women were enrolled. One participant later dropped midway into the study because of transportation difficulties. Seven women in total completed the study. The Institutional Review Board of the University of California at Los Angeles in accordance with assurances filed with and approved by the U.S. Department of Health and Human Services, approved the study, and participants provided written informed consent.

### Baseline and post intervention assessments

We conducted blood sampling, breast fluid collection, exercise testing, and anthropometry measurements in the week prior to starting the study. Once the last baseline measurement was made, patients were started the next day. We scheduled measurements to occur over a consecutive three-day period, with fasting hormone blood levels and anthropometric measurements taken on one day, exercise testing on another day, and ductal lavage procedures on the third day. Order of measurement days was random for each subject. Once the order of measurements was established at baseline, the same order was repeated at the end of the intervention, thereby minimizing influence of measurement order on the results. At the 12th week, measurements taken at baseline were repeated.

Body composition was assessed using the body-mass index measure (BMI), DEXA (dual energy x-ray absorptiometry) scanning, and Bioelectrical Impedance Analysis (BIA). BMI measurement included height assessment with a stadiometer and weight (mass) with a calibrated beam scale. To provide accurate measures of total body fat, whole body scans were given to subjects positioned supine on the DEXA scanning table (DEXA, GE Lunar Prodigy ® Advance 2006). The same licensed technician performed all scans. Bioelectrical impedance analysis (310e Bioimpedance Analyzer; Biodynamics, Inc, Seattle, WA) assessed BMR (basal metabolic rate) used to estimate baseline caloric intake for the dietary intervention.

### Exercise testing

An aerobic fitness assessment determined maximum oxygen consumption at baseline and at the end of the intervention. The maximum oxygen consumption (VO_2_ max) value was used to provide an intensity starting point for the aerobic exercise 12-week program undertaken for each of the participants. A maximum strength assessment determined strength at baseline and was used similarly to determine starting level for the resistance training regimen.

#### Testing for aerobic fitness

The VMax Encore®, Palm Springs, CA, designed to measure O_2_ and CO_2_ volumes utilized at rest and during exercise, monitored a 12-lead EKG, heart rate, and gaseous inhalation and exhalation. The graded exercise tolerance test was conducted with electrocardiogram monitoring to exclude individuals with subjective or objective evidence of coronary artery disease. The participants were sedentary. Therefore we started fitness assessment at the lowest exercise intensity ramp, and calibrated response to the ramp, with all subjects tested at baseline using the lowest ramp. The speed of the bicycle increased at one-minute intervals and continued increasing until subjects could no longer continue. The level at which they could no longer continue was measured by O_2_ consumption (VO_2_Max). All participants improved their fitness level sufficiently to ‘graduate’ to a higher ramp, and therefore we increased the ramp at the end of the intervention.

#### Testing for muscular strength

The ‘gold standard’ of dynamic strength testing is the 1-repetition maximum (1-RM). The 1-RM is the heaviest weight that can be lifted only once, using good form [30]. We conducted 1-Rep Maximum strength testing using the Brzycki formula [31] on calibrated air displacement weight equipment from Keiser®. The 1-Rep Maximum values were derived separately for the major muscle groups using a variety of weight machines that included Seated Leg Extension; Seated Chest Press; Seated Biceps Curl; Seated Triceps Pushdown; Seated Machine Row; Machine Squat; Seated Leg Press; and Hamstring Curl. Testing for 1-RM involved progressively increasing weight tension until participants reached their maximum exertion point.

### Ductal lavage

Ductal lavage involves the infusion of small amounts of sterile saline into a breast duct through a microcatheter where saline is infused into the duct and then the ductal effluent including the saline is collected. The procedure is commonly used to collect breast epithelial cells but can also be used to measure the endocrine microenvironment of the breast [28].

Ductal lavage was attempted immediately after nipple aspiration. Subjects were placed in the supine position. Skin in the nipple area was cleansed with 70% alcohol, and a fenestrated sterile drape was placed over the nipple. Ductal orifices were enlarged with dilators to facilitate cannulation. A separate microcatheter (available from Susan Love Foundation) was used for each duct cannulation to prevent cross-contamination between different individual ductal systems. After the microcatheter was inserted to a maximum depth of 1.5 cm, approximately 2 to 6 mL of normal saline was infused, and the breast compressed to facilitate recovery of ductal fluid into the collection chamber. This lavage procedure (infusion, compression and effluent collection) is repeated multiple times, instilling an average total volume of approximately 10 to 30 mL of normal saline and recovering approximately 5 to 20 mL of ductal effluent per duct. The exact infusion and effluent volumes was determined by weight to be used in the final calculations of the analytes. Location of each fluid-yielding duct and each cannulated duct was carefully marked on a 64-square nipple grid. The recovered ductal effluent was placed into tubes individually labeled for each cannulated duct. The effluent was spun at 3,000 rev for 10 minutes, the fluid transferred to aliquots, and frozen in a -80°C freezer.

We carefully recorded the breast we sampled and described the duct we cannulated at baseline, using the grid originally developed by Sartorius et al. (1977), so that we could return to the same duct at the 12th week of the intervention [5]. We limited our sampling to one duct per breast, and re-sampled the same duct from the same breast at the end of the intervention.

### Blood specimen collection

Blood was drawn into tubes after a 12 hour fast. We collected serum in tubes without heparin, and plasma and buffy coat in tubes with heparin. Serum, plasma and buffy coat were transferred to aliquots and frozen in a −80°C freezer.

### Laboratory measurement of serum and ductal lavage fluid

The study sample was small and all samples, both pre intervention and post intervention, were analyzed in the same batch. **Serum leptin** was determined by enzyme linked immuno assay (ELISA) from Diagnostic Systems Laboratory (Webster, TX). **Serum interleukin 6 (IL6)** was determined using the Quantikine® human immunoassay kit (R&D Systems Inc., Minneapolis, MN). **Serum estronesulfate** was determined by radioimmunoassay using a RIA (radioimmunoassay) assay kit (DSL-5400) from Beckman Coulter (Fullerton, CA), with a manufacturer determined intra-assay precision range of 9.2% for 0.35 ng/mL; 4.6% for 8.89 ngmL; and 4.7% for 59.33 ng/mL, and, our laboratory determined intra-assay precision of 6.5% for a concentration of 15 ng/mL. **Serum estradiol** concentration was determined using the Cayman EIA kit (Cayman Chemical, Ann Arbor, MI) (intra-assay precision of 15.8% for 41.0 pg/mL; 13% for 102.4 pg/mL; and 7.1% for 640 pg/mL, and a limit of sensitivity of 6.6 pg/mL(manufacturer-determined)). **Serum fatty acid analysis** was performed in serum hexane extracts. Fatty acids were converted to methyl esters (FAME) according to the method by Bagga et al. (1997) [32]. FAME were separated and quantified by use of an Agilent Technologies (San Diego, CA) 5890A series II gas chromatography fitted with a model 7673 automatic split-injection system and flame ionization detector and SP2380 stabilized phase fused silica capillary column (30 m × 0.32 mm i.d., 0.25 um film thickness, Supelco, Inc, Bellefonte, PA). Quantification was based on the recovery of a known quantity of the internal standard (tridecanoic acid, NuChek Preparation Inc., Elysian, MN) and on the response ratio of fatty acid standards purchased from NuChek Preparation Inc. (Elysian, MN). For quality control a pooled serum sample was used.

**Estradiol** concentration in ductal lavage fluid (DLF) was determined by gaschromatography mass spectrometry (GC-MS/MS) analysis as described by Zhang et al. (2006) [33]. 17β-estradiol (Sigma, E-2758), dissolved in methanol, was used to establish the standard curves. Deuterated estradiol (17β-estradiol-d3, Sigma #491187) was added as internal standard to DLF samples prior to column concentration. Samples were concentrated using the Supelco Discovery solid phase extraction DPA-6S columns (Supelco, Bellefonte, PA), pre-bis(trimethylsilyl)trifluoro-acetamide (BSTFA) with 1% trimethylchlorosilane (TMCS) catalyst (Supelco, Bellefonte PA,#3-3148) for derivatization at 65°C for 30 min. The derivatized samples were dried under a nitrogen stream and reconstituted with 50 μl hexane. Analyses were carried out using a ThermoQuest TRACE™ 2000 gas chromatography coupled with a ThermoQuest TRACE™ MS. Sample injection (1 μL) was in splitless mode. The GC column used was a Restek RTx-5 column (15 m × 0.25 μm × 250 μm). Helium carrier gas was maintained at a constant flow rate of 1.0mLmin − 1.

**Interleukin 6 (IL-6)** concentration in breast ductal fluid was determined using the Quantikine® human immunoassay kit (R&D Systems Inc., Minneapolis, MN).

### Description of the interventions

#### Dietary intervention

During the intervention period, patients were asked to consume only prepared meals distributed by the UCLA General Clinical Research Center (GCRC). Diets were comprised of 7 servings of fruits and vegetables, 20% fat, 30% protein, 50% carbohydrates, and 25–35 grams of fiber per day. Suggested caloric intake to achieve weight loss was based on a 500-calorie deficit of the participants’ basal metabolic rate (BMR) as determined by their BIA measurement conducted at the start of the study. BMR is derived from FFM (fat-free mass) using an equation by Grande et al. [34]. Base caloric level was established at 1200 calories per day.

Supplemental snacks, in addition to the three meal-per-day 1200 calorie regimen, tailored the intervention to each subjects’ BMR. All study subjects in the pilot diet and exercise intervention required snacks to supplement the 1200 calorie per day regimen, which suggested to us that the 1200 calorie baseline was a reasonable starting level to meet caloric requirements in the context of undergoing exercise training. Food was picked up from the GCRC by Center for Human Nutrition staff and distributed to study subjects twice per week. All participants received individual consultation on their respective diet plans with a registered dietitian throughout the study. Every four weeks (week 4 and week 8) subjects were weighed, and blood pressure and BMR measured.

#### Exercise intervention

Exercise training was custom-tailored to each woman’s strength and cardiovascular fitness. Participants began at an aerobic intensity that was 50% of their maximum oxygen uptake (VO_2_Max) determined from the VMax testing. We translated the VO_2_Max value into MET (metabolic equivalent of energy expenditure) units so that the corresponding intensity level for aerobic exercise could be determined [30]. Aerobic exercise occurred on treadmills and stationary bicycles. Weight training, beginning at 50% of the 1-repetition maximum (1-RM) recorded during muscular testing, was conducted using standard gym-based weight machines and free weights. Weight machines used in 1-RM testing were all available in the gym and were utilized along with supplemental free weights. At four week intervals, participants received updated exercises designed to increase their aerobic exercise by 10% of their VO_2_Max, and 10% of their 1-RM so that levels increased to 60%, 70% and 80% of their maximum values respectively.

Each participant met with the same exercise trainer for instruction using aerobic and weight resistance equipment at the designated exercise-training facility at UCLA, Fit Center South, for at least three times a week, for a minimum of one-hour sessions. Fit Center South was open 7 days a week during customary gym hours and was within close walking distance to the Center for Human Nutrition. On-site UCLA staff monitored subjects who use the exercise equipment. Notebooks contained each subject’s exercise routine. Subjects recorded their effort during their exercise intervention. Participants’ gym cards were scanned to validate attendance.

### Statistical analysis

Data were summarized with means and standard deviations calculated for continuous variables and frequencies for categorical variables using SAS 9.2 (Cary, NC). We computed percentage change relative to baseline and 95% confidence intervals for all exercise performance, body composition, and biomarker variables. Change in strength was summarized by averaging the 1-Rep Maximum values derived from the various Kaiser weight machines used for testing, and computing percentage change from baseline. Means are expressed with ± standard deviation (S.D.).

## Results

The seven women who participated in the study averaged 55 years old (55.3 ± 5.5 S.D.). Six were Caucasian with one Asian participant. Women weighed on average 89.8 kg ± 15.3 (197.9 pounds) at baseline. Participants were moderately obese, (average BMI of 33.6 kg/m^2^ ± 5.3), and had ‘low’ cardiovascular fitness [35,36] based on their VO_2_ Max measurements (13.8 ± 3.7) at baseline (see Table 1).

**Table 1:** **Mean body composition and exercise performance at baseline and post intervention**^**1**^

	**Baseline**		**Post intervention**		**Percent change**	
					**From baseline**	
**Variable**	**Mean**	**S.D.**	**Mean**	**S. D.**	**Mean**	**95% CI**
**Weight (kg)**	89.8	15.3	80.3	12.2	−10.3	(−12.6, -8.0)
**Body Mass Index (kg/m**^**2**^**)**	33.6	5.3	29.8	3.8	−11.0	(−13.9, -8.1)
**Fat Mass (kg)**^**2**^	41.3	11.9	35.5	10.9	−14.4	(−18.5, -10.3)
**Lean Mass (kg)**^**2**^	43.7	5.6	41.4	6.5	−5.4	(−11.1, 0.26)
**VO**_**2**_**Maximum (ml/kg/min)**^**3**^	13.8	3.7	19.0	6.3	36.1	(21.7, 50.5)
**1-REP Maximum (lbs)**^**4,5**^	103.5	25.7	130.3	36.8	25.9	(12.0, 39.8)

^1^ post intervention measurements occurred during the 12th intervention week.

^2^ measured by DEXA (dual-energy x-ray absorptiometry).

^3^ measured by VMax Encore®.

^4^ 1 repetition Maximum.

^5^ 1-REP Maximum was averaged over all the muscle groups tested.

We observed body composition and exercise performance improvements at the 12th intervention week compared to baseline. All subjects experienced reductions in BMI (average 11% reduction from baseline) and fat mass (14% reduction). Two subjects gained muscle mass, while the remaining five lost muscle mass, with an average overall muscle mass loss of 5%. Exercise performance improved from baseline. Average VO_2_Max increased by 36% and strength increased by 26%.

Estradiol and IL-6 were measured in ductal fluid at baseline and at the 12th week (see Table 2). Estradiol decreased 24% (from 10.5 ± 5.7 nmol/g protein to 8.1 ± 4.3 nmol/g protein) compared to baseline, while IL-6 changed 20% from baseline (0.5 ± 0.4 pg/mL to 0.4 ± 0.3 pg/mL).

**Table 2:** **Hormones, cytokines, and inflammatory factors contained in ductal fluid at baseline and post intervention**^**1**^

	**Baseline**		**Post intervention**		**Percent change**	
					**From baseline**	
**Variable**	**Mean**	**S.D.**	**Mean**	**S. D.**	**Mean**	**95% CI**
**Estradiol (nmol/g protein)**	10.5	5.7	8.1	4.3	−23.9	(−113.1, -10.5)
**IL-6 (pg/mL)**	0.5	0.4	0.4	0.3	−20.0	(−104.2, 72.2)

^1^ post intervention measurements occurred during the 12th intervention week.

We evaluated serum fatty acids, leptin, estrone-sulfate, estradiol, and IL-6 at baseline and at the 12th week of the intervention, while subjects were still undergoing the dietary and exercise regimen (see Table 3). We observed a 36% decline in serum leptin from baseline (dropping from 56.1 ± 26.4 ng/mL to 27.2 ± 20.1 ng/mL). Estradiol also decreased (24%) from baseline (157.9 ± 49.7 pmol/L dropped to 101.6 ± 27.9 pmol/L). Estrone-sulfate and IL-6 experienced declines from baseline (estrone sulfate dropped 10% from 5.8 ± 1.8 to 4.9 ± 2.8, and IL-6 dropped 33% from 2.3 ± 3.0 to 1.6 ± 2.7). Serum fatty acids were evaluated at the 12th week of the intervention while study subjects were still consuming the controlled dietary regimen. Total polyunsaturated fats increased slightly (5%) while total saturated fats decreased (5%) at the 12th week compared to baseline.

**Table 3:** **Mean serum hormones, cytokines, and fatty acids at baseline and post intervention**^**1**^

	**Baseline**		**Post intervention**		**Percent change**	
					**From baseline**	
**Variable**	**Mean**	**S.D.**	**Mean**	**S. D.**	**Mean**	**95% CI**
**Leptin (ng/mL)**	56.1	26.4	27.2	20.1	−35.5	(−76.1, -25.5)
**Estrone-Sulfate (nmol/L)**	5.8	1.8	4.9	2.8	−9.9	(−54.2, 34.3)
**Estradiol (pmol/L)**	157.9	49.7	101.6	27.9	−24.4	(−65.7, 17.0)
**IL-6 (pg/ml)**	2.3	3.0	1.6	2.7	−33.0	(−83.3, 8.3)
**Total Polyunsaturated Fats (% of total fats)**	43.9	6.1	45.5	2.3	5.3	(−7.3, 17.9)
**Total Saturated Fats (% of total fats)**	33.6	2.5	31.6	1.1	−5.4	(−13.1, - 2.2)

^1^ post intervention measurements occurred during the 12th intervention week.

## Discussion

The pilot study represents the first time hormone and cytokine biomarkers were measured in ductal fluid before and after a 12-week controlled dietary and exercise intervention. We observed reductions in estradiol and IL-6 levels contained in breast ductal fluid resulting from the intervention, suggesting a potential localization of changes to the breast environment as a function of the intervention.

Obese and sedentary women that lived in close proximity to UCLA were interested in the dietary and exercise intervention designed to promote breast cancer prevention as evidenced by their response to the web-based Love/Avon Army of Women invitation. We observed weight loss, fat mass loss, aerobic fitness and strength increases, and minimal muscle loss among our participants resulting from the intervention. The loss of muscle mass that we observed was consistent with other studies that included calorie restriction and exercise [37,38]. Ductal fluid sampling and measurement of hormones and cytokines contained within the fluid were both feasible.

Our intervention consisted of aerobic and resistance exercise in addition to calorie restriction. We could therefore not determine whether the fat mass loss and reduction in serum and ductal fluid estradiol occurred because of calorie restriction or exercise or both. Evidence from studies of premenopausal women suggest that both energy balance and nutritional status influence reproductive hormone levels [39]. We suspect that the fat mass loss, which occurred as a result of the intervention, was principally responsible for the reductions in serum and ductal fluid estradiol. However the caloric restriction and exercise could have also functioned to reduce estradiol independent of fat mass loss.

Several methods for localized breast sampling have been studied in the literature [40-43]. Sex steroid hormones in breast adipocytes were successfully measured in a small sample of 20 women undergoing breast clinical procedures [41]. While this procedure measured estradiol in digested adipose cells, it was unclear whether the breast fat estradiol reflected estradiol inside the breast ducts, although the evidence was suggestive. Nipple aspirate fluid (NAF) has been used in large cohort studies to assess risk by evaluating presence of NAF, cellularity of NAF, and whether atypical cells are present [42]. Postmenopausal women, in particular however, have lower yields of NAF than premenopausal women [43], and NAF sampling as a technique for collecting ductal fluid may not be possible for all postmenopausal women. We chose lavage because we could collect ductal fluid from non-NAF-fluid producing women [43], and because ductal fluid has been demonstrated to contain hormones, cytokines, and inflammatory factors in previous studies [26-28,44]. In our pilot study, three out of seven participants did not produce aspirate fluid when we conducted NAF before ductal lavage.

We preliminarily observed a reduction in estradiol contained in serum and breast ductal fluid suggesting that the fat mass loss may have promoted a reduction in aromatization to estradiol. In addition, the changes we observed systemically and locally suggest that the breast may be the recipient of two sources of estradiol. Chatterton et al. ( [2010]) examined patterns of serum steroid hormone level in premenopausal women compared to nipple aspirate hormone level in both pre- and postmenopausal women [44]. Whether the source of NAF estrogen was a result of biosynthesis from local androstenedione precursors or an enhanced rate of diffusion into the breast from blood could not be determined from their study or ours. We can however conjecture that postmenopausal women could potentially derive estrogen from two sources: adipose tissue aromatization occurring throughout the body, diffusing into the blood from the fat tissue, and transported to the breast; and, additionally, local diffusion of estrogen into the ducts from breast fat. Identifying the sources of estrogen to the breast will require a great deal of future research.

We observed in our pilot feasibility study a reduction in ductal fluid IL-6 and a reduction in serum IL-6. IL-6 present in ductal lavage fluid could reflect local inflammation at the breast [1,27] or systemic inflammation known to be linked to excess abdominal obesity [16]. The pattern of change we observed in IL-6 could be linked to the fat mass loss, particularly in the serum, but determining the source of IL-6 change was not possible.

Our results are preliminary and derived from a small sample that did not have controls. We established feasibility for conducting the diet and exercise intervention as well as demonstrating the capability to collect ductal samples and measure hormones and cytokines. The results are suggestive but not definitive.

## Conclusion

In summary, as a result of the pilot 12-week diet and exercise weight-loss intervention conducted among obese postmenopausal women, we observed systemic and localized reductions in serum and ductal fluid estradiol, and serum and ductal fluid IL-6.

## Abbreviations

VO_2_Max: Volume of maximal oxygen consumption; BMI: Body-mass index; DEXA: Dual energy x-ray absorptiometry; BIA: Bioelectric impedance analysis; FFM: Fat-free mass; IL-6: Interleukin 6; 1-RM: 1 repetition maximum; DLF: Ductal lavage fluid; ELISA: Enzyme-linked immunoassay; RIA: Radio immunoassay; FAME: Fatty acid methyl esters; GCRC: General clinical research center; BMR: Basal metabolic rate.

## Competing interests

The authors declare that they have no competing interests.

## Authors’ contributions

CLC conceived of and participated in the research design, conducted and coordinated the research, analyzed the data, and drafted the manuscript. KD participated in research design and conduct. PJ designed and implemented the dietary intervention. LL participated in biomarker laboratory analysis. SH designed the biomarker assays and participated in laboratory analysis. ZL participated in design and conduct of the research. DH participated in research design and helped to draft the manuscript. All authors read and approved the final manuscript.
